The article "Expression of Inflammatory Factors in Critically Ill Patients with Urosepticemia and the Imaging Analysis of the Severity of the Disease" was retracted in 2023. Reasons: signs of a paper mill; suspected computer-generated content; unreliable results or conclusions; lack of ethics approval or compliance.

# Expression of Inflammatory Factors in Critically Ill Patients with Urosepticemia and the Imaging Analysis of the Severity of the Disease

**DOI:** 10.1155/2021/6659435

**Published:** 2021-02-20

**Authors:** Xia Huang, Zongjun Hu, Xi Yue, Yong Cui, Jiwen Cui

**Affiliations:** Department of Critical Care Medicine Neurosurgery, Chongqing University Three Gorges Hospital, Wanzhou, Chongqing 404000, China

## Abstract

Urine sepsis is a complex inflammatory response of the body to infection with a high fatality rate. It is one of the main causes of death in noncardiovascular intensive care units. Nevertheless, in daily clinical practice, early sepsis is often not detected. In this paper, discharged cases of urinary sepsis from the Department of Urology and Critical Care Medicine of a university hospital were collected as the observation group, and common urinary tract infection cases were selected as the control group. We sorted and summarized the discharged case information of the observation group and the control group. The results of the study showed that, after renal pelvis perfusion, the expression of HMGB1 protein and mRNA increased, and the expression of TLR4 increased; inhibiting HMGB1 can reduce the expression of inflammatory factors caused by perfusion and reduce the infiltration of neutrophils and macrophages caused by perfusion. In addition, r HMGB1 treatment can promote the expression of inflammatory factors caused by perfusion and aggravate the infiltration of neutrophils and macrophages caused by perfusion. We found that inhibition of HMGB1 can inhibit the expression of TLR4/My D88 signaling molecules and r HMGB1 treatment can enhance the expression of TLR4/My D88 signaling molecules.

## 1. Introduction

Urinary calculi are a very common clinical disease. In recent years, the clinical incidence of this disease in my country has shown an upward trend [1]. At present, percutaneous nephrolithotomy (PNL) has become the first treatment for urinary system stones, especially stones with longest diameter ≥ 20 mm and complicated structures [2, 3]. PNL has the clear advantages of ideal curative effect and direct effect. With its wide application, various postoperative complications have gradually received extensive clinical attention [4]. The incidence of postoperative complications of PNL can reach about 29% to 80%. Postoperative fever can easily induce severe complications such as renal function damage and kidney loss [5]. If timely and effective treatment is not given, it may even progress to urinary sepsis, which endangers the life of the patient. Therefore, it is clear that the related factors and independent risk factors for urosepsis after PNL and corresponding prevention and treatment before and after surgery can effectively reduce the incidence of urosepsis after surgery, ensure the efficacy of surgery, and improve the quality of patient prognosis [6, 7].

The article "Expression of Inflammatory Factors in Critically Ill Patients with Urosepticemia and the Imaging Analysis of the Severity of the Disease" was retracted in 2023. Reasons: signs of a paper mill; suspected computer-generated content; unreliable results or conclusions; lack of ethics approval or compliance.

Urinary calculi are a frequently occurring disease in clinical practice. In recent years, the incidence has gradually increased. With the continuous development and improvement of medical microendoscopy technology and the gradual maturity of minimally invasive technology, PCNL has become the first choice for the treatment of urinary stones, especially large stones, complex, and specific stones, and it has ideal clinical effects [8, 9]. However, postoperative complications of PNL are still an important part of surgical treatment that cannot be ignored. The clinical incidence of fever after PNL is about 25.8% to 39.8%, of which about 0.3% to 4.7% can progress to urinary sepsis, which can induce septic shock and multiple organ failure (MODS) to endanger patients' safety of life [10]. Therefore, it is necessary to conduct in-depth analysis and research on relevant clinical data to clarify the risk factors of urosepticemia after PNL and to provide a basis and ideas for adjuvant treatment of PNL in the future. Elderly patients aged 60 years and above are more likely to have symptoms of urosepticemia after surgery, which are mainly related to the patients' own basic diseases and the decline of various body functions [11]. The anatomy of the female urethra is one of the main reasons why women are susceptible to urinary tract infections, and after menopause, the level of estrogen in the body drops significantly, which reduces their physical resistance [12]. Therefore, female patients are more likely to develop urosepsis after PNL. The mucosal tissue of the renal pelvis is the body barrier against bacterial invasion, and the operation time is prolonged. The larger the volume of the stone during the operation is, the more the fragments will be after the lithotripsy [13]. The risk of damage to the renal pelvic mucosa will increase, and the opening time of blood vessels will be prolonged. In order to promote the discharge of gravel and maintain the clarity of the surgical field, the intraoperative perfusion must be increased. The increase in the contact surface of the perfusate with the tissue will increase the absorption [14]. The gravel and inflammatory tissues are under high pressure. The perfusion fluid flows back into the blood, thereby increasing the risk of postoperative infection. Therefore, the probability of postoperative urosepsis will increase. Patients with upper ureteral calculi are more likely to have a fever after surgery. The main reason is that the upper ureteral obstruction can form hydronephrosis, which increases the risk of infection and may even form empyema, which causes bacteria to enter the blood through the damaged renal pelvic mucosa during the operation [15–17]. At the same time, the upper ureteral calculi can aggravate the inflammatory reaction and the difficulty of the operation and induce postoperative urosepticemia. It has been reported that 51.5% of urinary tract infections will develop fever, 31.9% will develop urosepsis, 2% will develop severe sepsis, 0.3% will develop septic shock, and the mortality rate is as high as 30%–50%. Studies have reported that C-reactive protein (CRP) has a good negative predictive effect, so it can be used for the diagnosis of SIRS and urosepsis excretion. CRP will increase 4 to 6 hours after bacterial infection and double at a rate of 8 hours, peaking at 36–50 hours after infection, and its plasma half-life is 19 hours. In the acute infection period, its level can reach between several hundred times and several thousand times the normal value, but its value will also decrease after the cause is eliminated. In macrophages, the combination of HMGB1 and TLR4 occurs in the early stages of inflammation [18, 19]. We found that HMGB1 can regulate the activation of the TLR4 signaling pathway in the kidney after high-pressure perfusion. Using neutralizing antibodies to inhibit HMGB1 can significantly reduce the expression of TLR4 signaling pathway-related proteins while adding recombinant HMGB1 to the perfusion fluid has the opposite effect [20–22].

The article "Expression of Inflammatory Factors in Critically Ill Patients with Urosepticemia and the Imaging Analysis of the Severity of the Disease" was retracted in 2023. Reasons: signs of a paper mill; suspected computer-generated content; unreliable results or conclusions; lack of ethics approval or compliance.

Decreased renal blood flow and renal insufficiency can make it difficult for antibiotics to reach the infected lesion and cannot neutralize endotoxins. Therefore, urinary sepsis may still occur after routine preoperative antibiotics to prevent infection. Early removal of obstruction can protect residual renal function, thereby helping to control infection. Specifically, the technical contributions of this paper can be summarized as follows.

First, before surgery, we routinely indwell urine culture and give sensitive antibiotic anti-infection treatment based on the urine culture drug sensitivity result, which can kill some pathogenic bacteria, but prolonged use of antibiotics may also lead to the production of conditional pathogens. Changshi can cause urinary sepsis.

Second, all the obstructive patients included in this study were able to gradually improve after the obstruction was relieved through conventional treatment and were discharged smoothly. After high-pressure perfusion, the expression of HMGB1 increases, and the expression of inflammatory factors increases, accompanied by inflammatory cell infiltration.

The article "Expression of Inflammatory Factors in Critically Ill Patients with Urosepticemia and the Imaging Analysis of the Severity of the Disease" was retracted in 2023. Reasons: signs of a paper mill; suspected computer-generated content; unreliable results or conclusions; lack of ethics approval or compliance.

Third, studies have shown that HMGB1 neutralizing antibody can significantly reduce the inflammatory response caused by the rapid increase in renal pelvic pressure. Therefore, HMGB1 antibody administered during the perioperative period of PNL may attenuate the inflammatory response. HMGB1 neutralizing antibody has been proven to reduce inflammation in animal ischemic injury models. Studies have shown that adding recombinant HMGB1 to the perfusion fluid can aggravate the inflammatory response after renal pelvic hypertension.

The rest of this paper is organized as follows.  Section 2 discusses the high-risk factors of urosepticemia and the diagnosis and treatment of critically ill patients.  Section 3 gives information and methods.  Section 4 analyzes the experimental results.  Section 5 summarizes the full text.

## 2. High-Risk Factors of Urosepsis and Diagnosis and Treatment of Critically Ill Patients

### 2.1. High-Risk Factors and Common Causes of Urosepticemia

Urinary tract infection is an inflammatory response of the urothelium to bacterial invasion, often accompanied by bacteriuria and pyuria. More than 50% of women have had urinary tract infections in their lives; about 10% of men over 60 have experienced asymptomatic bacteriuria. In patients with long-term indwelling catheters in clinical practice, the presence of bacteria will be found in urine routine. Pathogens can invade the genitourinary system through the upper and lower urinary tract, blood, lymphatic channels, and so on. Whether it causes urinary tract infection is closely related to the number, virulence, and defense barrier of the body. Under normal circumstances, pathogenic bacteria that enter the body are quickly cleared by the body's immune system. Risk factors such as advanced age, history of diabetes, urinary tract obstruction, and urinary calculi can cause the spread of infection and cause a series of clinical symptoms. If not diagnosed and treated in time, it quickly progresses to serious urinary system infections. Critically ill patients can develop hemodynamic disturbances and shock, which can lead to serious complications such as multiple system dysfunction. Early diagnosis and active treatment are the keys to control urosepsis and reduce the mortality rate.

Symptoms and signs are the main basis for the diagnosis of urinary tract infection. Symptoms such as changes in body temperature, dysuria, frequent urination, urgency, and suprapubic pain are often the only symptoms of early urinary tract infection. These clinical manifestations are often not obvious in people with low immunity, so clinical manifestations are used as the basis for early diagnosis. Among them, vital signs are a general indicator, and continuous dynamic monitoring has certain clinical significance, but the specificity of early diagnosis of serious infections such as urosepsis is not high.

The article "Expression of Inflammatory Factors in Critically Ill Patients with Urosepticemia and the Imaging Analysis of the Severity of the Disease" was retracted in 2023. Reasons: signs of a paper mill; suspected computer-generated content; unreliable results or conclusions; lack of ethics approval or compliance.

Bacterial culture is recognized as the gold standard for the diagnosis of urinary tract infections at home and abroad. During clinical operation, not all bacterial cultures of patients with urinary tract infection can accurately reflect the status of bacteria. The results are affected by the body's immunity and the recent application of antibiotics. In the early stage of urinary tract infection, there are fewer bacteria, excessive fluid intake, or urine dilution caused by catheterization, which will cause false-negative results in urinalysis and urine culture. The positive rate of clinical urinary system bacterial culture is low, and the culture result is lagging. Although it has guiding value for clinical treatment, it has poor timeliness. Most patients with urinary tract infection have symptoms of bladder irritation. The urine enters the bladder and is excreted quickly. Pathogens do not have enough time to multiply, the concentration is low, and the diagnostic threshold is not reached, resulting in low urine culture colony counts. Therefore, bacterial culture should be combined with other biochemical detection indicators and clinical symptoms for comprehensive diagnosis and treatment. The schematic diagram of the role of TSP-1 in inflammation is shown in Figure 1.

In clinical work, blood routine, urine routine, CRP, and other inflammatory indicators are the main monitoring methods. The abnormal percentage of neutrophils in routine blood tests can indicate the presence of urinary tract infections, but the specificity of disease diagnosis is low, and other diagnostic indicators need to be combined to determine the site of infection, and the value of determining the severity of infection is limited. The test results of each group in this study showed that the percentage of neutrophils was generally increased, and the severity of urinary tract infection was related to the age of the patients. When severe sepsis or shock occurred, some patients had neutrophils. The percentage of routine blood NEU and the increase in routine urine WBC count indicate inflammation in the body. These two indicators are not statistically different in the comparison between the urea sepsis group and the urea sepsis complicated shock group. The early diagnosis of the disease has limited value. Drawing the ROC curve also shows that the area under the curve of routine blood NEU% and urine routine WBC count is small, which lacks the accuracy of the diagnosis of urosepsis.

The article "Expression of Inflammatory Factors in Critically Ill Patients with Urosepticemia and the Imaging Analysis of the Severity of the Disease" was retracted in 2023. Reasons: signs of a paper mill; suspected computer-generated content; unreliable results or conclusions; lack of ethics approval or compliance.

With the increase of age, the body's immune system will degenerate. The immune system participates in the body's inflammatory response and plays an important role in fighting diseases. Its aging indicates the decline of disease resistance. Older patients are more susceptible to infections, and the disease is more difficult to control, which is a risk factor for the worsening of severe urea sepsis.

### 2.2. Analysis of the Etiology of Urosepticemia during the Treatment of Upper Urinary Tract Stones by Minimally Invasive Intracavitary Surgery

With the development of intracavitary urology, minimally invasive surgery such as endoscopy basically replaces most of the traditional open surgery in urology, especially urinary calculi. Urinary sepsis caused by urinary surgery is probability of occurrence in clinical work.

Surgical time is an independent influencing factor for postoperative complications of urosepticemia. Urinary endoscopic surgery is different from traditional open surgery. In order to maintain a clear vision during the operation, continuous lavage under certain water pressure and long-term continuous irrigation are required. Washing can cause increased pressure on the renal pelvis. Intraoperative renal pelvic pressure increases (>30 mm Hg), which will cause reflux in the renal pelvis, which may cause postoperative fever and sepsis. In one case, the double J tube was twisted and reflexed after the operation, and effective drainage was not obtained. Renal endotoxin was absorbed continuously, and the infection was difficult to be effectively controlled. After another operation to adjust the position of the double J tube, the sepsis was quickly controlled. One case underwent second-stage percutaneous nephrolithotomy without a drainage tube during the operation. Sepsis occurred after the operation. The analysis of the cause may also be related to the poor drainage of the urine after the operation. To analyze and summarize the above, it can be preliminarily considered that surgical methods, uncontrolled preoperative infections, complexity of stones, long operation time, delayed anesthesia resuscitation, and postoperative drainage are related to the high-risk factors for postoperative infection of urosepsis.

The urinary system is connected to the outside world through the urethra. Under normal circumstances, due to the continuous washing of urine and the defense effect of the urethral mucosa, bacteria are not easy to stay and multiply in the urethra for a long time and are not easy to be infected. For patients with urinary system obstruction, urine drainage is not smooth, providing a growth environment for bacteria, while the obstruction of the urinary system leads to increased pressure in the renal pelvis and acute damage to renal function. Bacteria and endotoxins enter the blood circulation through various return routes and cause infection. However, many patients have a rapid onset and rapid progress. At this time, it is often difficult for antibacterial drugs to reach effective drug concentration in the infected lesions, and the effect of anti-infection treatment alone is often not good. While actively fighting infections and correcting the overall condition, surgical drainage should be actively used to relieve obstruction, drain urine, and protect kidney function. At this time, the patient's condition is often severe, and surgery with relatively large surgical trauma is not suitable. The two commonly used surgical methods in this group of patients include ureteroscopic ureteral stent placement under local anesthesia and percutaneous nephrostomy. Relieving the obstruction at the time is the key to treatment, and the cause can be completely relieved in the second stage. The schematic diagram of the pathogenesis mediated by immune-inflammatory cells and factors is shown in Figure 2.

The article "Expression of Inflammatory Factors in Critically Ill Patients with Urosepticemia and the Imaging Analysis of the Severity of the Disease" was retracted in 2023. Reasons: signs of a paper mill; suspected computer-generated content; unreliable results or conclusions; lack of ethics approval or compliance.

For patients with urinary obstruction, early active surgical drainage to relieve the obstruction has a significant effect on infection control and treatment, improving the progress of the disease, shortening the treatment time of sepsis, and reducing the mortality rate.

### 2.3. Selection of Surgical Drainage Methods

There were no operative complications in ureteroscopic ureteral stent implantation, and there was no significant difference between the two in statistics (*p* > 0.05). In terms of the control time of urosepticemia, the control time of ureteroscopic ureteral stent implantation is 3.9 ± 1.6 days, while the control time of percutaneous nephrostomy is relatively short, 3.6 ± 1.4 days. It is considered that it may be relatively larger than the percutaneous nephrostomy tube with more thorough drainage and not easy to block. However, there was no statistically significant difference between the two (*p* > 0.05). It can be seen that the two surgical methods have no significant differences in the treatment of sepsis, infection control, success rate, complications, and treatment time. Compared with clinicians, ureteroscopic stent placement has relatively low clinical technical requirements, which can be mastered by low-age clinicians. Unsuccessful catheter placement under ureteroscopy is often due to severe obstruction of the stone and extreme distortion of the ureter. Percutaneous nephrostomy requires B-ultrasound real-time positioning, certain requirements for ultrasound technology, and needs to penetrate the kidney, there is a certain risk of bleeding, and the difficulty is easily affected by renal hydrops.

The article "Expression of Inflammatory Factors in Critically Ill Patients with Urosepticemia and the Imaging Analysis of the Severity of the Disease" was retracted in 2023. Reasons: signs of a paper mill; suspected computer-generated content; unreliable results or conclusions; lack of ethics approval or compliance.

When the diameter of hydronephrosis is more than 2 cm, percutaneous nephrostomy is safer and more successful. For patients with thrombocytopenia and coagulopathy, ureteroscopic stent placement is also the priority. Regarding the choice of single J tube and double J tube, double J tube is most commonly used in clinic, but the lumen of double J tube is relatively small, which is easy to block for cloudy and thick urine or pus. If the urine is cloudy and thick, or when the kidney is purulent, and if the hydronephrosis is not obvious or the coagulation function is severely impaired, percutaneous nephrostomy should not be performed. At this time, a single J tube can be considered. External flushing to replace turbid urine or pus is effective, or after flushing and replacing urine, it can be externally drained or replaced with a double J tube, but whether it will increase the probability of ascending infection needs further study. Of course, for patients with obvious purulent kidney or perirenal infection and obvious hydronephrosis but no obvious coagulation dysfunction, they are more inclined to undergo percutaneous nephrostomy because the lumen of the fistula is relatively larger, not easy to be blocked, and even if blocked after the operation, it can be flushed and recanned at low pressure. Ureteroscopic ureteral stent placement and percutaneous nephrostomy are both safe and effective for emergency treatment of ureteral stone obstruction with sepsis, but the success rate of ureteral stent placement under ureteroscope is higher; for unskilled surgeons and patients with mild hydronephrosis, ureteroscopy is recommended. There is no significant difference in the success rate and safety of the two surgical methods, but the time of percutaneous nephrostomy in the treatment of urosepsis is relatively short. The cavity is larger and the drainage is smoother.

Considering that, with the development of the medical level in recent years, people's in-depth research on sepsis and the standard and emphasis on clinical treatment and the development and application of advanced medical equipment have led to a trend of lower overall mortality. For patients with urinary tract obstruction, while fighting infection in the early stage, surgical drainage is actively used to relieve the obstruction. When a patient fails to actively surgical drainage due to various reasons in the early stage and serious complications occur, such as patients with extremely reduced platelets and shock, we are actively fighting shock and supplementing platelets, and we also actively draining the patients, resulting in mortality.

The article "Expression of Inflammatory Factors in Critically Ill Patients with Urosepticemia and the Imaging Analysis of the Severity of the Disease" was retracted in 2023. Reasons: signs of a paper mill; suspected computer-generated content; unreliable results or conclusions; lack of ethics approval or compliance.

## 3. Materials and Methods

### 3.1. Clinical Data

For the diagnostic criteria of urinary tract infection, see the 2014 Chinese Urological Disease Diagnosis and Treatment Guidelines, with bladder irritation symptoms such as frequent urination, urgency, painful urination, hematuria, back pain, and costal and spinal angle tenderness, while meeting one or more of the following conditions: ① urine sediment microscopic examination showing urine white blood cell count > 5HPF; ② nitrite positive or urine white blood cell esterase positive; ③ clean midsection urine bacterial culture ≥ 10^5^/ml.

For diagnostic criteria of urinary sepsis, see the 2014 Chinese Urological Diseases Diagnostic and Treatment Guidelines. Diagnostic criteria of urinary sepsis are induced by urinary tract infection, with 2 or more of the following items: ① body temperature > 38°C or <36°C; ② heart rate > 90 beats/min; ③ respiration rate > 20 beats/min or arterial blood carbon dioxide partial pressure < 32 mm Hg or mechanical ventilation; ④ peripheral blood white blood cell count > 12 × 10^9^/L or <4 × 10^9^/L or immature white blood cells > 10%.

The diagnostic criteria for urinary sepsis meets the following two conditions at the same time: ① urinary tract infection: one or more of the following conditions are met: urine white blood cell count > 5HPF; nitrite positive; urine leukocyte esterase positive; pus in the celiocentesis fluid or pus moss in the stones; ② in line with systemic inflammatory response syndrome, see the Western medicine diagnostic criteria for details.

Case exclusion criteria are as follows:

(1) Severe heart, brain, liver, and kidney diseases, such as heart failure, severe liver, and kidney failure; (2) congenital malformations such as abnormal anatomy of the urinary system, polycystic kidney, horseshoe kidney, or obstruction of the junction of the kidney and ureter; (3) accompanied by hematological diseases, antitumor therapy, oral immunosuppressive drugs, and other immune-dysfunction diseases or mental disorders; (4) combined with other systemic infectious diseases.

### 3.2. Research Methods

Cases of urinary sepsis which met the inclusion criteria were taken as the observation group; cases with urinary tract infection and nonsepticemia were taken as the control group.

This study adopted a retrospective research method. A total of 45 diagnosed cases of urinary sepsis were collected and observed within the observation period. Four cases were excluded and excluded, including 1 case with bladder malignant tumor, 2 cases with bleeding after PCNL operation, and severe 1 case of renal failure; 41 eligible cases were collected.

The article "Expression of Inflammatory Factors in Critically Ill Patients with Urosepticemia and the Imaging Analysis of the Severity of the Disease" was retracted in 2023. Reasons: signs of a paper mill; suspected computer-generated content; unreliable results or conclusions; lack of ethics approval or compliance.

We select the occurrence of inflammatory response syndrome (SIRS) as the onset time node of the included cases and record the body temperature, respiration, heart rate, and blood pressure at the onset and peripheral blood white blood cell counts within 6 hours, 12 hours, 24 hours, 3 days, and 7 days after the onset (WBC), neutrophil count (NEU), procalcitonin (PCT), CRP, brain natriuretic peptide (BNP), coagulation function (including PT, APTT, and FIB), and D-dimer body.

In addition, we collect discharged cases of nonurinary sepsis and urinary tract infection during the observation period (control group) and record their hospitalization number, gender, age, basic conditions, WBC, NEU, PLT, PT, APTT, FIB, and other related indicators.

The SPSS 22.0 statistical software package was used for statistical data processing, and all continuous variables passed the normal distribution test and the homogeneity of variance test. Two independent-sample *t*-tests were used for comparison between two groups, one-way analysis of variance was used for comparison between three or more groups, and LSD (*L*) was used for pairwise comparison; nonparametric test was used for measurement data that did not conform to the normal distribution. *p* < 0.05 indicates that the difference is statistically significant. The data of the four-grid table adopt the chi-square test. The technical route studied is shown in Figure 3.

### 3.3. Diagnostic Laboratory Indicators of Urinary Sepsis

The incidence of sepsis continues to rise, the mortality rate is high, and early diagnosis is the key to the diagnosis and treatment of sepsis. Observing the early specific and sensitive blood indicators of urinary sepsis has important clinical significance. Early warning of urinary sepsis can effectively reverse the progression of the disease and reduce the risk of death. At present, the commonly used laboratory indicators of sepsis are as follows.

#### 3.3.1. Procalcitonin (PCT)

PCT is a precursor protein of calcitonin, consisting of 116 amino acid residues. The PCT content in normal human serum is < 0.05 ng/ml. Under normal circumstances, PCT is secreted by thyroid C cells, and its concentration in the blood is relatively stable. When irritated by severe trauma, major surgery, and severe infection, PCT is produced by other organs outside the thyroid, such as liver, lung, kidney, and adrenal gland, and released into the blood circulatory system. The PCT begins to increase within 2–4 hours after the body is infected by bacteria, reaches a peak at 6–8 hours, and maintains a high level at 8–24 hours, with a half-life of 25–30 hours. As an indicator of inflammation, PCT is closely related to the severity of infection. PCT is significantly increased in the blood of patients with systemic infection, while there is no change or only a slight increase in the blood of patients with mild or local infection; in sepsis, PCT is always at a high level. The dynamic changes of PCT can indicate the prognosis of sepsis. If the PCT declines after treatment, the prognosis is good, and if it continues to rise, the prognosis is poor. Compared with other inflammatory indicators such as CRP, IL-6, IL-8, and white blood cells, PCT has certain advantages in the early auxiliary and differential diagnosis of sepsis and the judgment of disease severity, efficacy, and prognosis.

The article "Expression of Inflammatory Factors in Critically Ill Patients with Urosepticemia and the Imaging Analysis of the Severity of the Disease" was retracted in 2023. Reasons: signs of a paper mill; suspected computer-generated content; unreliable results or conclusions; lack of ethics approval or compliance.

#### 3.3.2. BNP and N-Terminal Precursor Brain Natriuretic Peptide (NT-pro-BNP)

BNP is a neuropeptide synthesized by ventricular myocytes. When ventricular pressure or volume increases, myocardial cell expansion prompts the body to release active BNP and inactive NT-pro-BNP, which can reflect heart function. The elevated levels of plasma BNP and pro-BNP in patients with septic shock are mainly related to myocardial depression and cardiac insufficiency.

#### 3.3.3. White Blood Cells and Neutrophils

When bacteria invade, white blood cells are the body's first line of defense and have nonspecific immune effects. They are produced in the bone marrow through the action of colony-stimulating factor (G-CSF) and released to the peripheral blood circulation. Studies have shown that blood leukocytes and neutrophils are the first to change in urinary sepsis after PCNL, and even before clinical manifestations and vital signs change, the level of leukocytes or neutrophils drops sharply. For the characteristic of change, white blood cells are mostly less than 3 × 10^9^/L and neutrophils are mostly less than 2 × 10^9^/L. In the upper urinary tract lithotripsy, a large amount of endotoxin is released into the blood, producing a large number of inflammatory factors, triggering a systemic inflammatory response, a large number of white blood cells enter the interstitial space, and the white blood cells and neutrophils in the peripheral blood decrease. Therefore, monitoring the change trend of white blood cells and neutrophils after intracavitary lithotripsy has certain clinical significance for predicting urinary septic shock. However, WBC is used to diagnose bacterial infections with low accuracy and low specificity. Some physiological and infectious factors can cause it to rise. Systemic infections can lead to an increase in WBC or a decrease in WBC, which has certain limitations.

#### 3.3.4. CRP and Hypersensitive CRP

CRP is an acute phase protein synthesized by liver cells when the body is subjected to inflammatory stimuli such as bacterial infection or tissue damage. When there is inflammation or infection, serum CRP can rise rapidly in a short period of time, which can promote the body's complement system to exert nonspecific immune function, so it is a nonspecific anti-inflammatory factor. The CRP level of sepsis patients was higher than that of nonsepticemia patients (*p* < 0.05), and the serum CRP level of sepsis death group was higher than that of survival group (*p* < 0.05). However, CRP has high sensitivity and low specificity, and it has certain limitations as a monitoring indicator of sepsis. hs-CRP is a CRP detected by an ultrasensitive method. It is more sensitive to the diagnosis of bacterial infectious diseases than CRP and is one of the nonspecific markers reflecting SIRS. The diagnostic efficiency of hs-CRP in diagnosing sepsis is second only to PCT. It begins to increase at 12–18 hours after sepsis infection, reaches a peak at 24–48 hours, and continues to peak at 1–3 days after infection. After inflammation is cleared, its content dropped sharply and could return to normal within 1 week. Therefore, CRP and hs-CRP as nonspecific inflammatory indicators can differentiate between bacterial infection and nonbacterial infection, help early diagnosis of sepsis, and have certain predictive significance for the severity and prognosis of the disease.

The article "Expression of Inflammatory Factors in Critically Ill Patients with Urosepticemia and the Imaging Analysis of the Severity of the Disease" was retracted in 2023. Reasons: signs of a paper mill; suspected computer-generated content; unreliable results or conclusions; lack of ethics approval or compliance.

#### 3.3.5. Serum Lactic Acid and Lactic Acid Clearance Rate

Blood lactic acid can reflect tissue hypoxia. When the patient has severe sepsis or septic shock, the body is damaged by inflammation, the whole body or local tissues have poor blood perfusion, and the oxygen supply of organs and tissues is insufficient, which cannot meet the needs of body tissue metabolism, resulting in continuous accumulation of arterial blood lactic acid content. With the progress of sepsis, liver failure, the liver's ability to clear lactic acid continues to decrease, the content of lactic acid in the body gradually increases, and the damage to the body is aggravated, resulting in a vicious circle. Arterial blood lactic acid at admission has an important role in evaluating the condition and prognosis of elderly patients with severe sepsis and septic shock. However, the general basic conditions of patients are different, and their response to stress is also different. Simply monitoring the blood lactic acid concentration at a certain moment cannot accurately reflect the condition and treatment effect. Therefore, some people have suggested that it should be more scientific to use lactic acid clearance rate to dynamically monitor blood lactic acid.

Existing treatment methods have improved the cure rate of sepsis to a certain extent, such as fluid resuscitation, broad-spectrum and sensitive antibiotics, mechanical ventilation, glucocorticoids, intensive insulin therapy, recombinant human activated protein, blood transfusion, plasma, and continuous blood purification treatment. At present, for the treatment of urinary sepsis, the following four strategies are mainly recommended: ① Stabilize blood pressure and maintain unobstructed breathing through resuscitation and support treatment. ② Use empirical, broad-spectrum antimicrobial treatment as early as possible, especially in sepsis-induced hypotension within 1 hour. ③ Control the concomitant factors, such as urinary tract obstruction, and use ureteroscope or cystoscope retrograde placement of double “J” tube drainage and percutaneous renal puncture fistula. Toxemia is treated to control the infection, and further surgery is performed after the condition is stable. ④ Use special treatments, such as the application of hydrocortisone to patients with a relatively insufficient function of the pituitary-adrenal cortex axis and the application of insulin to strictly control blood sugar. However, the mortality rate of severe sepsis and septic shock is still high, indicating that there are still deficiencies. Sepsis treatment has become the biggest obstacle to further improving the success rate of critically ill treatment. Early diagnosis is the key to treating sepsis. Clinically, early diagnosis of sepsis and timely antibiotic treatment can reduce the mortality rate. Therefore, how to early and accurately predict and diagnose sepsis and implement reasonable treatment measures is the key to improving the survival rate of sepsis.

The article "Expression of Inflammatory Factors in Critically Ill Patients with Urosepticemia and the Imaging Analysis of the Severity of the Disease" was retracted in 2023. Reasons: signs of a paper mill; suspected computer-generated content; unreliable results or conclusions; lack of ethics approval or compliance.

## 4. Experimental Results and Analysis

### 4.1. The Effect of Renal Pelvic Hypertension on the Expression of HMGB1

At different time points after renal pelvic hypertension, Western blot and q RT-PCR were used to detect the expression of HMGB1 protein and m RNA in kidney tissues. As shown in Figure 4, after the renal pelvis is perfused with high pressure, the expression level of HMGB1 protein gradually changes and reaches its peak at 3 h after perfusion. In addition, the level of HMGB1 m RNA also has a similar trend. In short, after renal pelvic hypertension perfusion, HMGB1 protein expression and m RNA expression levels increased.

### 4.2. The Effect of Renal Pelvic Hypertension on the Expression of Inflammatory Factors

Through the animal PCN model, the effect of renal pelvic hypertension perfusion on the level of inflammatory factors in kidney tissue was studied. As shown in Figure 5, the mRNA levels of the inflammatory factors TNF-*α*, IL-1*β*, and IL-6 in the kidney tissue reached a peak 6 hours after perfusion and then gradually declined.

The article "Expression of Inflammatory Factors in Critically Ill Patients with Urosepticemia and the Imaging Analysis of the Severity of the Disease" was retracted in 2023. Reasons: signs of a paper mill; suspected computer-generated content; unreliable results or conclusions; lack of ethics approval or compliance.

At all monitored time points after perfusion, the expression of IL-1*β* at 21 h after perfusion was significantly higher than the expression of inflammatory factors TNF-*α* and IL-6 in the serum.

### 4.3. Inhibition of HMGB1 on the Inflammatory Response Caused by Renal Pelvic Hypertension

In order to study the effect of HMGB1 on the expression of inflammatory factors caused by increased renal pelvic pressure after PCN, this paper uses HMGB1 neutralizing antibody to inhibit HMGB1. As shown in Figure 6, the addition of HMGB1 neutralizing antibody to the perfusion fluid can significantly inhibit the mRNA expression levels of inflammatory factors TNF-*α*, IL-1*β*, and IL-6, while the addition of control antibody to the perfusion fluid does not affect the inflammatory factors mRNA expression level.

The expression of serum inflammatory factors TNF-*α*, IL-1*β*, and IL-6 was inhibited by the neutralizing antibody of HMGB1, while the control antibody treatment was not affected. In order to observe the expression of inflammatory factors in kidney tissue, this paper uses IHC to detect the expression of inflammatory factors at 4 h after perfusion. The imaging results of immunohistochemical detection of inflammatory factors in kidney tissue are shown in Figure 7.

### 4.4. The Effect of HMGB1 Treatment on the Inflammatory Response Caused by Renal Pelvic Hypertension

In order to further study the effect of HMGB1 on the expression of inflammatory factors caused by high-pressure renal pelvic perfusion, recombinant HMGB1 was added to the perfusion fluid to analyze the mRNA expression levels of inflammatory factors 4 hours after perfusion. The results in Figure 8 show that r HMGB1 treatment can increase the mRNA expression level of inflammatory factors.

As shown in Figure 9, through the kidney tissue IHC, we found that r HMGB1 treatment can significantly aggravate the infiltration of neutrophils and macrophages caused by high-pressure perfusion.

## 5. Conclusion

Urinary sepsis is often insidious, with many interfering factors. Urinary tract infections are common, and stone obstruction is more common. Patients are often admitted to the hospital with renal colic and urinary tract infection. Early diagnosis is the key to the treatment of urinary sepsis. Inflammation indicators are more sensitive than coagulation indicators in diagnosis. It may be that abnormal coagulation function is activated by inflammation. The coagulation reaction is only promoted when the inflammatory response damages the endothelial cells to a certain extent. Therefore, the inflammation indicators often appear abnormal before the coagulation indicators, and they are more serious. The coagulation function is obviously abnormal only after infection or even septic shock, so inflammation indicators have higher sensitivity. This study found that the HMGB1/TLR4 signaling pathway plays an important role in the occurrence of urosepsis after percutaneous nephroscopy in hypertensive renal pelvic perfusion. HMGB1 can induce inflammation through the TLR4 signaling pathway. HMGB1 neutralizing antibody can suppress this inflammation, while recombinant HMGB1 can aggravate the inflammatory response. The results of this study will help prevent inflammation caused by increased renal pelvic pressure during PNL. One limitation of this study is that it did not detect changes in renal function, so it is impossible to know the influence of HMGB1 mediated inflammation on renal pathology. In future studies, this paper will examine the related renal function of animal PCN models after treatment with HMGB1 neutralizing antibody and recombinant HMGB1, such as the detection of serum creatinine levels and urine output, in order to prevent and treat postoperative inflammatory reactions.

The article "Expression of Inflammatory Factors in Critically Ill Patients with Urosepticemia and the Imaging Analysis of the Severity of the Disease" was retracted in 2023. Reasons: signs of a paper mill; suspected computer-generated content; unreliable results or conclusions; lack of ethics approval or compliance.

## Figures and Tables

**Figure 1:** Schematic diagram of the role of TSP-1 in inflammation.

**Figure 2:** Schematic diagram of pathogenesis mediated by immune-inflammatory cells and factors.

**Figure 3:** Technical route of research.

**Figure 4:** q RT-PCR detection of HMGB1 m RNA level in kidney tissue.

**Figure 5:** q RT-PCR detection of mRNA expression levels of inflammatory factors in renal tissues at different time points after renal pelvic hypertension perfusion.

**Figure 6:** q RT-PCR detection of mRNA expression levels of inflammatory factors in kidney tissue after inhibiting HMGB1 treatment.

**Figure 7:** Imaging analysis of the expression of inflammatory factors in renal tissue detected by immunohistochemistry.

**Figure 8:** q RT-PCR detection of mRNA expression levels of inflammatory factors in renal tissues after r HMGB1 treatment.

**Figure 9:** Immunohistochemical detection of inflammatory cell infiltration in the interstitium of renal tissue. (a) Neutrophil, irrigation + PB. (b) Neutrophil, irrigation + r HMG. (c) Macrophage, irrigation + PB. (d) Macrophage, irrigation + r HMG.

## Data Availability

The data used to support the findings of this study are available from the corresponding author upon request.
